This article has been retracted.

# MicroRNA‐320a inhibits invasion and metastasis in osteosarcoma by targeting cytoplasmic polyadenylation element‐binding protein 1

**DOI:** 10.1002/cam4.2919

**Published:** 2020-02-17

**Authors:** Yanlong Wang, Jiyu Yang, Pangtao Chen, Yu Song, Weizheng An, Haoran Zhang, Butegeleqi Butegeleqi, Jinglong Yan

**Affiliations:** ^1^ Departments of Orthopedic Surgery The Second Affiliated Hospital of Harbin Medical University Harbin Heilongjiang P.R. China

**Keywords:** cytoplasmic polyadenylation element‐binding protein 1, microRNAs, miR‐320a, osteosarcoma

## Abstract

Osteosarcoma is a primary malignant bone tumor, which affects children, adolescents, and young adults commonly. MicroRNAs (miRNAs) have been proved to be dysregulated in different cancers, including osteosarcoma. Although miR‐320a has been implicated in many types of malignancies, little is known about the role of miR‐320a in osteosarcoma. In this study, we show that the overexpression of miR‐320a or knockdown of cytoplasmic polyadenylation element‐binding protein 1 (CPEB1) inhibited osteosarcoma cell migration and invasion. miR‐320a downregulates CPEB1 expression by directly targeting the CPEB1 3′‐UTR. Furthermore, CPEB1 reintroduction reversed the antiproliferation, antimigration, and antiinvasion roles of miR‐320a, indicating that miR‐320a might function as a tumor suppressor in osteosarcoma through CPEB1. In conclusion, our study demonstrates that miR‐320a plays a critical role in osteosarcoma progression and may provide a potential therapeutic target for osteosarcoma.

## 1 INTRODUCTION

Osteosarcoma is a primary malignant bone tumor^1^, ^2^, ^3^ and affects children, adolescents, and young adults commonly and occurs mostly in the distal femur, proximal tibia and humerus.^3^, ^4^, ^5^ The swelling in the affected bone and onset of pain are the typical presentation of osteosarcoma and the pain could wake patients from sleep.^6^, ^7^ Approximately 18% of patients can detect metastases clinically at presentation and most of the metastatic disease occurs in the lung, and bones are the second most common site of metastatic disease.^8^, ^9^ Although treatment for osteosarcoma advances from amputation to complex limb‐sparing surgeries and pharmacological agents, many patients fail to respond.^10^ Therefore, it is an emergency to identify the mechanism of osteosarcoma occurrence and development and effective therapeutic approaches for osteosarcoma.

MicroRNAs (miRNAs) are endogenous non‐coding small RNAs (18‐25 nt) which modify gene expression at transcriptional and posttranscriptional levels in eukaryotic cells.^11^, ^12^, ^13^ About 3% of human genes code for endogenous miRNAs synthesis and more than 32% of human genes can be regulated by miRNAs.^14^, ^15^, ^16^ A number of biological processes are regulated by miRNAs, including cell development, embryogenesis, cell maintenance, and lineage determination.^17^, ^18^, ^19^, ^20^ miRNAs have been reported to perform an increasingly pivotal role in human diseases. Studies have shown that miRNAs participate in liver cancer, neurodegenerative disease, cardiovascular disease, and other diseases.^21^, ^22^, ^23^, ^24^ Increasing evidence has also shown that miRNAs play an important role in osteosarcoma progression.^25^, ^26^, ^27^, ^28^ For example, miRNA‐21 was found upregulated in osteosarcoma tissues and cells and inhibition of miRNA‐21 could inhibit osteosarcoma cell proliferation.^29^ miR‐1284 was proved to be a new regulator to inhibit osteosarcoma cell proliferation and migration.^30^

miR‐320a was previously proved as a tumor suppressor in many cancers such as colorectal cancer^31^ and hepatocellular carcinoma.^32^ However, the biological role and clinical function of miR‐320a in osteosarcoma is still unknown. Therefore, in this study, we investigated the function of miR‐320a in osteosarcoma cells. We found that upregulated miR‐320a inhibited cell growth ability in vitro and in vivo and inhibited cell migration, and invasion. miR‐320a regulates osteosarcoma by targeting cytoplasmic polyadenylation element‐binding protein 1 (CPEB1). Our findings will provide new insights into the molecular function of miR‐320a in osteosarcoma and hopefully provide a potential therapeutic target for osteosarcoma.

## 2 MATERIALS AND METHODS

### 2.1 Mouse experiments

Male athymic BALB/c nu/nu mice used in these experiments (aged 4 weeks) were purchased from Shanghai Laboratory Animal Center (Shanghai, China). All animal experiments were in accordance with the Care and Use of Laboratory Animals which was published by the US National Institutes of Health. For mice injection, 7 × 10^6^ U2OS cells transfected with miR‐320a mimic or CPEB1 siRNA and the control cells were injected subcutaneously into the right flank of the nude mice. The size of tumors was measured every 3 days. After 20 days, the mice were sacrificed and photographed and tumor weight was measured finally. Eight mice were included in each group.

### 2.2 Cell lines and culture conditions

Two osteosarcoma cell lines (143B and U2OS) were cultured with RPMI‐1640 medium (GIBCO, USA) and supplemented with 10% fetal bovine serum (FBS) (Aidenbach, Germany) and antibiotics (100 U/mL penicillin G and 100 μg/mL streptomycin, GIBCO). Human osteoblast cells (hFOB) were cultured with dulbecco's modified eagle medium (DMEM)/F12 medium (GIBCO) and supplemented with 10% FBS and antibiotics. The three cell lines were purchased from the Shanghai cell bank of Chinese Academy of Sciences and were cultured at 37°C in a humified incubator with 5% CO_2_.

### 2.3 miRNAs, siRNAs and cell transfection

The primers for miR‐320a mimics 5′‐AAA AGC UGG GUU GAG AGG GCG A‐3′(sense), 5′‐GC CCU CUC AAC CCA GCU UUU UU‐3′ (antisense), CPEB1 siRNA 5′‐CCAAGCTTCCAATATCTTTCGAAGGATAAATGC‐3′ (sense) and 5′‐GGCCGTCGACAAGTCA‐ GACCCAAGGGGATCCAGAG‐3′(antisense) negative control RNA duplex: 5′‐UGA AUU AGA UGG CGA UGU UTT‐3′ (sense), 5′‐AAC AUC GCC AUC UAA UUC ATT‐3′(antisense) were synthesized by AMBiotech. miR‐320a inhibitor and its negative control were obtained from AMBiotech. Cells were seeded into a six‐well plate and when the cells grown to 60%‐80% confluency, transfected the cells using Lipofectamine 2000 (Invitrogen), according to the manufacturer's protocols.

### 2.4 Quantitative real‐time PCR analysis (qRT‐PCR)

Total RNA was isolated using TRIZOL reagent (Invitrogen) according to the manufacturerʼs protocol. qRT‐PCR was employed to determine the mRNA expression of miR‐320a and CPEB1. qRT‐PCR was performed using SYBR Green qPCR Master Mix (TAKARA). The primer sequences are as follows. miR‐320a (F: 5′‐AAA AGC TGG GTT GAG AGG GCG A‐3′; R: 5′‐GCG AGC ACA GAA TTA ATA CGA C‐3′) and U6 snRNA (F: 5′‐CTC GCT TCG GCA GCA CA‐3′; R: 5′‐AAC GCT TCA CGA ATT TGC GT‐3′). U6 was used for normalization. CPEB1 (F: 5′‐CCTGGGTATTAGCCGACAGT‐3′); R: 5′‐GCCTCAGCATTTAGCATTCC‐3′) and GAPDH (F: 5′‐TTG TTG CCA TCA ATG ACC C‐3′; R: 5′‐CTT CCC GTT CTC AGC CTT G‐3′). β ‐catenin: (F: 5′‐ ATGGAGCCGGACAGAAAAGC‐3′, R: 5′‐ CTTGCCACTCAGGGAAGGA‐3′); aquaporins 1: (F: 5′‐GAC‐ ACCTCCTGGCTATTGACTACA‐3′; R: 5′‐CCGCGGAGCCAAAGG‐3′); aquaporins 4: (F: 5′‐ AGCCTGGGATCCACCATC‐3′R: 5′‐TGCAATGCTGAGTCCAAAGC‐3′). Heat‐shock protein 20: (F: 5′‐ GAGTGGGACTGAAGGAAATGG‐3′R: 5′‐ATCTTGGGGTTGTCACTGGC‐3′). GAPDH was used for normalization. All primers were obtained from AMBiotech.

### 2.5 3‐(4,5‐Dimethylthiazol‐2‐yl)‐2,5‐ diphenyltetrazolium bromide assay (MTT assay)

The two cell lines were seeded in 96‐well culture plates at a density of 10 000 cells per well. When the cells reached 60‐80% confluence, they were transfected with the required oligonucleotide. After transfection for 24, 48, or 72 hours, the cells were stained with 20 μL of MTT (5 mg/mL), (Sigma) for 4 hours at 37°C. The cell medium was carefully aspirated and 150 μL of dimethyl sulfoxide was added to each well. Then, the absorbance at 490 nm was measured.

### 2.6 Colony formation assay

For colony formation ability, 143B and U2OS cells were transfected with miR‐320a mimic, miR‐320a inhibitor, or NC and subsequently seeded in 6‐cm plates at a concentration of 1 000 cells/dish and incubated in the incubator to allow for colony formation. After 2 weeks, the colonies were fixed using methanol. Then, the colonies were stained with 0.1% crystal violet (Sigma) and counted.

### 2.7 Migration and invasion assay

For the cell migration assay, the cells were seeded in the transwell unit with 8‐μm polycarbonate nucleopore filters (Corning Costar). The upper chamber contained serum‐free medium and the medium in lower compartment contained 10% FBS; the cells were kept in the incubator for 24 hours. The cells in the lower surface of the filter were fixed and calculated. For the cell invasion assay, the membrane of the transwell unit was coated with 40 μL Matrigel (BD, USA) at 37°C for 4.5 hours to form a basement membrane and the cells were treated in a similar fashion as that in the cell migration assay.

### 2.8 Western blotting analysis

Total cells or tissue extracts were extracted using cell lysis buffer followed by immunoblotting with anti‐CPEB1 (CST, USA). Cells were lysed in ice‐cold radio‐immunoprecipitation assay (RIPA) buffer with protease inhibitors (Roche Applied Science) on ice for 30 minutes and then centrifuged for 20 minutes at 13 500 rpm at 4°C. The supernatant was transferred to a new Eppendorf tube and the protein concentration was measured using a BCA protein assay kit (Applygen). Thirty micrograms of cell lysates was resolved with 12.5% sodium dodecyl sulfate polyacrylamide gel electrophoresis and transferred to nitrocellulose membranes. Then, the membranes were blocked with 5% skim milk for 2 hours at room temperature (RT). After blocking, the membranes were incubated with primary antibody at 4°C overnight. Then the membranes were washed, and incubated with secondary antibodies at RT for 1 hour. The protein bands were visualized using ECL reagent (HaiGene, China). Protein bands were analyzed using ImageJ 1.61 software.

### 2.9 Luciferase reporter assay

The CPEB1 3′‐UTR was cloned into pGL3 luciferase reporter (Promega), generating pGL3‐ CPEB1.

QuikChange Site‐Directed Mutagenesis Kit (Stratagene) was used to introduce mutations in potential miR‐320a binding sites. One microgram of miR‐320a mimic or its control was cotransfected with 1 μg constructs into U2OS cells. The dual‐luciferase reporter assay was performed after 24 hours using the Dual‐Luciferase Reporter Assay Kit (Promega) according to the manufacturer's protocol.

### 2.10 Statistical analysis

Data are presented as mean ± standard deviation (SD), and the experiment was repeated at least three times. Statistical differences were assessed by one‐way analysis of variance (ANOVA) or two‐way ANOVA. Statistical differences were considered when *P < .05.

## 3 RESULTS

### 3.1 miR‐320a inhibits osteosarcoma cell proliferation in vivo and in vitro

To investigate the role of miR‐320a in osteosarcoma progression, we measured the expression of miR‐320a in osteosarcoma cells (Figure 1A) and compared with hFOB cells, the expression of miR‐320a was downregulated in 143B and U2OS cells. MTT assay was performed with two osteosarcoma cell lines 143B and U2OS, which had been transfected with miR‐320a mimic or the negative control (NC) mimic (Figure 1B). These data indicated that the overexpressed miR‐320a inhibited osteosarcoma cell proliferation ability in 143B and U2OS cells (Figure 1C,D). After the expression of endogenous miR‐320a was silenced by miR‐320a inhibitor, the proliferation ability in the two cell lines increased (Figure 1E,G). Moreover, colony formation assay was performed. Decreased proliferation ability was found in miR‐320a overexpressed cells compared with control and increased growth ability was found in miR‐320a inhibited cells compared with the control (Figure 2A,B). These data indicate that miR‐320a inhibited osteosarcoma cell proliferation ability in vitro.

**Figure 1:** miR‐320a inhibits cell proliferation ability in vitro. A, Relative miR‐320a expression levels in hFOB, 143B and U2OS cells were detected using qRT‐PCR. B, Relative miR‐320a expression levels in 143B and U2OS cells were detected using qRT‐PCR after transfection with the miR‐320a mimic or its control (NC mimic). C and D, MTT assays were performed with 143B (C) and U2OS (D) cells after transfection with the NC mimic or the miR‐320a mimic. E, Relative miR‐320a expression levels in 143B and U2OS cells were detected using qRT‐PCR after transfection with miR‐320a inhibitor and negative control (NC inhibitor). F and G, MTT assays were performed with 143B (F) and U2OS (G) cells after transfection with miR‐320a inhibitor or NC inhibitor. The experiments were independently repeated three times. (*P < .05; **P < .01; ***P < .001)

**Figure 2:** miR‐320a inhibits osteosarcoma cell proliferation in vivo and in a xenograft model. A and B, Colony formation assays. 143B and U2OS cells were transfected with NC mimic or miR‐320a mimic and NC inhibitor or miR‐320a inhibitor. C, Tumors formed in nude mice. 7 × 10^6^ U2OS cells transfected with NC mimic or miR‐320a mimic and NC inhibitor or miR‐320a inhibitor were subcutaneously injected into the nude mice (n = 8). The mice were then sacrificed 20 days after the injection. Representative tumor images are shown. D, The tumor volumes were measured. E, Tumors and the bodies were weighted and the data are expressed as tumor weight (TW)/body weight (BW). F, Scatter graph of tumor weight and each dot represents the tumor weight of each mouse. The experiments were independently repeated three times. (*P < .05; **P < .01; ***P < .001)

To examine the function of miR‐320a in osteosarcoma cell proliferation ability in vivo, a xenograft model of osteosarcoma cells was applied to nude mice. U2OS cells were transfected with miR‐320a mimic or its control and then he transfected cells were injected into the cortex of the anterior tuberosity. A significant decrease was observed in tumor weight and size of miR‐320a overexpressed groups when compared with its control groups (Figure 2C‐F). U2OS cells transfected with miR‐320a inhibitor or its control were injected into the cortex of the anterior tuberosity of the nude mice and the tumor weight and size were increased compared with NC inhibitor (Figure 2C). All these results show that miR‐320a significantly inhibited osteosarcoma cell proliferation ability.

### 3.2 Osteosarcoma cell migration and invasion are inhibited when miR‐320a is overexpressed

qRT‐PCR was performed to confirm the overexpression of miR‐320a in 143B and U2OS cells transfected with miR‐320a mimic (Figure 3A). Then transwell assays with or without Matrigel were performed. The without Matrigel transwell assays demonstrated that the miR‐320a mimic group significantly suppressed the migration of 143B and U2OS compared with the control (Figure 3B,C). The with Matrigel transwell assays showed that invasion ability was significantly decreased in 143B and U2OS cells transfected with miR‐320a mimic. (Figure 3D,E). The U2OS cells transfected with miR‐320a inhibitor or NC inhibitor were supplied with transwell assays with or without Matrigel (Figure 3F). The without Matrigel transwell assays demonstrated that the miR‐320a inhibitor group significantly promoted the migration of U2OS compared with the control (Figure 3G,H). The with Matrigel transwell assays showed that invasion ability was significantly increased in U2OS cells transfected with the miR‐320a inhibitor group. (Figure 3G,H). These results show that miR‐320a overexpression inhibits osteosarcoma cell migration and invasion.

**Figure 3:** Overexpression of miR‐320a inhibits 143B and U2OS cells migration and invasion. A, 143B and U2OS cells were transfected with NC mimic or miR‐320a mimic and were confirmed using qRT‐PCR. B, Representative image of 143B and U2OS cells migration. D, Representative image of 143B and U2OS cell invasion. C and E, Quantitative results of migration and invasion cell numbers of 143B and U2OS cells. The experiments were independently repeated three times. (*P < .05; **P < .01; ***P < .001). F, 143B and U2OS cells were transfected with NC inhibitor or miR‐320a inhibitor and were confirmed using qRT‐PCR. G, Representative image of U2OS cells migration and invasion. H, Quantitative results of migration and invasion cell numbers of U2OS cells. The experiments were independently repeated three times. (*P < .05; **P < .01; ***P < .001)

### 3.3 miR‐320a regulates the expression of CPEB1 by targeting the 3′‐UTR of CPEB1 directly

To identify the potential targets of miR‐320a, bioinformatics strategies were used. The CPEB1 3′‐UTR that was predicted on TargetScan had one target site for miR‐320a (Figure 4D). We measured the expression of CPEB1 in hFOB, 143B and U2OS cells using western blot and CPEB1 was upregulated in 143B and U2OS cells compared with hFOB cells (Figure 4A). Western blot and qRT‐PCR results (Figure 4C,F) showed that miR‐320a overexpression suppressed the mRNA and protein levels of CPEB1 in 143B and U2OS cells. The luciferase reporter assay was performed to investigate whether miR‐320a regulates CPEB1 by targeting the 3′‐UTR of CPEB1 directly. The luciferase reporter assay results showed a significantly decreased luciferase activity in pGL‐ CPEB1‐3′UTR compared with its control groups, but the mutated effective target reporter was not repressed by miR‐320a (Figure 4E). Moreover, we measured the expression of β‐catenin, aquaporins 1, aquaporins 4 and heat‐shock protein 20 using qRT‐PCR after transfection with miR‐320 mimics, which have been proven to be the genes downstream of miR‐320a. However, no apparent change was observed between NC mimics and miR‐320 mimic groups (Figure 4G). These results show that miR‐320a targeted the 3′UTR of CPEB1 directly and regulated CPEB1 expression.

**Figure 4:** miR‐320a directly targets the CPEB1 3′‐UTR. A and B, Western blotting was performed to detect the protein expression levels of CPEB1 in hFOB, 143B and U2OS cells. C and F, qRT‐PCR and western blotting were performed to detect the mRNA and protein expression levels of CPEB1 in the 143B and U2OS cells transfected with the NC mimic or miR‐320a mimic. D, The prediction targeting site of CPEB1 3′‐UTR combined with miR‐320a are shown. E, HEK‐293T cells were cotransfected with wild‐type 3′‐UTR (WT) or mutant‐type 3′‐UTR (MT) reporters and the NC mimic or the miR‐320a mimic. In the experiments shown in the panels, luciferase/Renilla activity was measured. G, qRT‐PCR was performed to detect the mRNA levels of β‐catenin, aquaporins 1, aquaporins 4 and heat‐shock protein 20. The experiments were independently repeated three times. (*P < .05; **P < .01; ***P < .001)

### 3.4 Downregulated CPEB1 inhibits osteosarcoma cell proliferation ability and metastasis

143B and U2OS cell lines were transfected with CPEB1 siRNA or its negative control. Western blot and qRT‐PCR were performed to confirm the transfection efficiency in 143B and U2OS cells transfected with CPEB1 siRNA or its negative control (Figure 5A,B) and then MTT assays and transwell assays were performed. The MTT assay (Figure 5C,D) results show that silencing of CPEB1 expression inhibited the proliferation ability of 143B and U2OS cells. The transwell assay (Figure 5E‐H) results also showed a decrease of migration and invasion ability in 143B and U2OS cells. U2OS cells transfected with CPEB1 siRNA or its negative control were injected into nude mouse and the results show that the size and weight of tumors in CPEB1 siRNA groups was significantly decreased (Figure 6A‐E). All these data show that downregulated CPEB1 inhibits osteosarcoma cell proliferation ability and metastasis.

**Figure 5:** CPEB1 downregulation inhibits the proliferation and migration of osteosarcoma cells. A and B, The 143B and U2OS cells were transfected with negative control (siNC) and CPEB1 siRNA (siCPEB1). The mRNA level and protein level of CPEB1 after interference were detected using qRT‐PCR and western blotting. C and D, 143B and U2OS cells were applied to MTT assay after transfection of siNC and siCPEB1. E and G, The transwell assays with and without Matrigel were performed in 143B and U2OS cells transfected siNC and siCPEB1. F and H, Quantitative results of migration and invasion cell numbers of 143B and U2OS cells. The experiments were independently repeated three times. (*P < .05; **P < .01; ***P < .001)

**Figure 6:** CPEB1 is involved in miR‐320a decreased growth and migration in osteosarcoma cells. A, Tumors formed in nude mice. The U2OS cells transfected with CPEB1 siRNA and its control were subcutaneously injected into eight nude mice. B, The volumes of formed tumors were determined. C, Tumors and the bodies were weighted and are shown as tumor weight (TW)/ body weight (BW). D, Representative mRNA level of CPEB1 in tumor tissues. E, Scatter graph of tumor weight and each dot represents the tumor weight of each mouse. F, 143B and U2OS cells were cotransfected with miR‐320a mimics and its negative control (NC), miR‐320a mimics plus the empty vector (miR‐320a + pc3.0), miR‐320a mimics plus the CPEB1 overexpression vector (miR‐320a + pc3.0 + CPEB1). G. 143B and U2OS cells were cotransfected with miR‐320a inhibitor and its negative control (In‐NC), and miR‐320a inhibitor plus the siRNA against CPEB1 (In‐ miR‐320a + siCPEB1). The expression of CPEB1 was detected using qRT‐PCR. H‐K. The cells transfected as in (F and G) were used for transwell assays. L and M MTT assays were performed with the cells transfected as in (F and G). The experiments were independently repeated three times. (*P < .05; **P < .01; ***P < .001)

### 3.5 CPEB1 is involved in miR‐320a regulated proliferation and migration in osteosarcoma cells

143B and U2OS cell lines were transfected with miR‐320a mimic (miR‐320a) or its control NC or miR‐320a plus the empty vector (miR‐320a + pc3.0), or miR‐320a + pc3.0 plus the CPEB1 overexpression vector (miR‐320a + pc3.0 + CPEB1), or miR‐320a inhibitor (In‐ miR‐320a) or its control In‐NC, or In‐ miR‐320a plus CPEB1 siRNA (In‐ miR‐320a + siCPEB1), respectively. qRT‐PCR results showed that miR‐320a inhibited CPEB expression (Figure 6F,G). Transwell and MTT assays results showed that restoration of CPEB1 increased miR‐320a‐induced suppression of osteosarcoma cell proliferation (Figure 6L,M), migration (Figure 6H,I) and invasion (Figure 6J,K). These data show that miR‐320a targeted CPEB1 and inhibited osteosarcoma cell growth and migration partially through CPEB1.

## 4 DISCUSSION

Osteosarcoma arises from osteoid tissue and is one of the most common primary sarcoma of bone and produces immature bone.^33^ Osteosarcoma occurs in adolescents most frequently and can be found at the end of long bones usually, which is a leading cause of cancer death among adolescents and young adults.^34^, ^35^ Since the huge economic pressures on osteosarcoma patients and their families, it is emergency to identify the mechanism of osteosarcoma development and establish new strategies for osteosarcoma treatment. Previous studies indicate that miRNAs dysregulation may affect epigenetic information and may be considered to play a significant role in the pathogenesis of osteosarcoma.^36^, ^37^ Therefore, identification of osteosarcoma‐associated miRNAs and its clinical significance and functions may provide a missing piece of osteosarcoma.

miR‐320a is encoded in the antisense orientation of the cell cycle gene POLR3D and plays a critical role in transcriptional silencing expression of POLR3D.^38^, ^39^, ^40^ Many studies have proved that miR‐320a could inhibit cell proliferation, induces apoptosis, affect cell cycle and plays a critical role of anti‐tumor in many cancers.^41^, ^42^, ^43^, ^44^ However, the relationship between expression of miR‐320a and osteosarcoma progression remains unclear.^45^, ^46^, ^47^ So, we hypothesized that miR‐320a affects the proliferation and development of osteosarcoma in this research. MTT assays and colony formation assay results show that miR‐320a overexpression inhibited osteosarcoma cells’ proliferation ability in vitro and the results of tumor formation in nude mice show that miR‐320a overexpression inhibited osteosarcoma cells proliferation ability in vivo. To investigate the function of miR‐320a in osteosarcoma, transwell assays were performed and the results show that miR‐320a inhibited cell migration and invasion of osteosarcoma, indicating that miR‐320a inhibits osteosarcoma development through cell proliferation, migration, and invasion ability.

A growing body of studies showed that there are many down‐stream target genes of miR‐320a. In 2012, Sun et al showed that miR‐320a could directly target β‐catenin to suppress the growth of colon cancer cells.^48^ Sepramaniam et al in 2010 proved that the precursor miR‐320a functions as an inhibitor of aquaporin 1 and 4 expression but anti‐miR‐320a functions as an activator of aquaporin 1 and 4 expression. Treatment with anti‐miR‐320a could reduce the infarct volume in cerebral ischemia along with increased expression of aquaporin 1 and 4.^49^ Recent studies have identified a critical role of miR‐320a in the regulation of cardiomyocyte death. Cardiomyocyte death and apoptosis were enhanced when miR‐320 was overexpressed and treatment with antagomir‐320 in vivo reduced infarction size; Ren et al identified heat‐shock protein 20 as an important target for miR‐320 in these processes using proteomic analysis and TargetScan software.^50^

Cytoplasmic polyadenylation element‐binding protein (CPEB) plays a key role in mRNA translation, which binds the 3′‐UTRs of responsive mRNAs in cytoplasmic polyadenylation element.^51^, ^52^ CPEB1 is a dual‐function protein in Xenopus oocytes.^53^, ^54^ A close correlation between CPEB1 and cancers has been demonstrated and high expression levels of CPEB1 in tumor cell lines have also been shown.^55^, ^56^ In this study, we validated that CPEB1 was a direct target of miR‐320a and the protein and mRNA level of CPEB1 was shown to be decreased when miR‐320a was overexpressed, indicating a negative correlation between miR‐320a and CPEB1 expression in osteosarcoma. MTT assay and transwell assay results show that CPEB1 downregulation inhibited the proliferation and migration of osteosarcoma cells and the results of tumors formation in nude mice showed the same data pattern. To further strengthen our data, the MTT and transwell assays were performed to show whether the restoration of CPEB1 could increase miR‐320a‐induced suppression of cell proliferation, migration and invasion and the results show that CPEB1 is involved in miR‐320a decreased proliferation ability and migration in osteosarcoma cells. In conclusion, our research shows that miR‐320a functions as a tumor suppressor in osteosarcoma by targeting CPEB1. These results indicate that miR‐320a might regulate the expression of CPEB1 during the development and progression of osteosarcoma. These results give us a novel insight that miR‐320a regulates osteosarcoma by potentially targeting CPEB1. Our finding provides new insights into the molecular function of miR‐320a in osteosarcoma and hopefully may provide a potential therapeutic target for osteosarcoma.

## CONFLICT OF INTEREST

The authors declare that they have no conflict of interest.

## AUTHOR CONTRIBUTION

Yanlong Wang and Jinglong Yan designed the experiments; Yanlong Wang, Jiyu Yang and Pangtao Chen carried out the experiments; Yanlong Wang analyzed experimental results. Yu Song, Weizheng An and Haoran Zhang analyzed the sequencing data and developed the analysis tools. Butegeleqi assisted with Illumina sequencing. Yanlong Wang and Jinglong Yan wrote the manuscript.

## Data Availability

The datasets used during this study are available from the corresponding author on request.
